The article "Multi-dimensional perceptual recognition of tourist destination using deep learning model and geographic information system" was published in 2025. Journal: PLoS One.

# Multi-dimensional perceptual recognition of tourist destination using deep learning model and geographic information system

**DOI:** 10.1371/journal.pone.0318846

**Published:** 2025-02-07

**Authors:** Shengtian Zhang, Yong Li, Xiaoxia Song, Chenghao Yang, Niusha Shafiabady, Robert M. X. Wu

**Affiliations:** 1 School of Computer and Network Engineering, Shanxi Datong University, Datong, China; 2 School of Architecture, Tsinghua University, Beijing, China; 3 Department of Information Technology, Peter Faber Business School, Australian Catholic University, Sydney, Australia; 4 Faculty of Engineering and Information Technology, University of Technology Sydney, Sydney, Australia; Sakarya University: Sakarya Universitesi, TÜRKIYE

## Abstract

Perceptual recognition of tourist destinations is vital in representing the destination image, supporting destination management decision-making, and promoting tourism recommendations. However, previous studies on tourist destination perception have limitations regarding accuracy and completeness related to research methods. This study addresses these limitations by proposing an efficient strategy to achieve precise perceptual recognition of tourist destinations while ensuring the integrity of user-generated content (UGC) data and the completeness of perception dimensions. We integrated various types of UGC data, including images, texts, and spatiotemporal information, to create a comprehensive UGC dataset. Then, we adopted the improved Inception V3 model, the bidirectional long short-term memory network (BiLSTM) model with multi-head attention, and geographic information system (GIS) technology to recognize basic tourist feature information from the UGC dataset, such as the content, sentiment, and spatiotemporal perceptual dimensions of the data, achieving a recognition accuracy of over 97%. Finally, a progressive dimension combination method was proposed to visualize and analyze multiple perceptions. An experimental case study demonstrated the strategy’s effectiveness, focusing on tourists’ perceptions of Datong, China. Experimental results show that the approach is feasible for studying tourist destination perception. Content perception, sentiment perception, and the perception of Datong’s spatial and temporal characteristics were recognized and analyzed efficiently. This study offers valuable guidance and a reference framework for selecting methods and technical routes in tourist destination perception.

## Introduction

Tourist perceptions of the destination convey behavioral, psychological, emotional, and attitudinal information. Recognizing the perception of a tourist destination is an effective way to reveal the image and personality of the destination and serves as an essential guide for potential visitors [1–3]. Furthermore, the practical and precise recognition of tourist perception of the destination is vital for promoting the development of tourist destinations and making recommendations.

The article "Multi-dimensional perceptual recognition of tourist destination using deep learning model and geographic information system" was published in 2025. Journal: PLoS One.

Previous studies recognized the perceived content from the tourist questionnaire and achieved high accuracy through qualitative analysis. However, some problems were observed in the data sampling and analysis, such as labor, high time costs, and data limitations [4, 5]. Recently, user-generated content (UGC) has emerged as more users interact through online platforms. People use online social media platforms, such as Flickr, TripAdvisor, and Sina Weibo, to reflect their perceptions of destinations through text, photos, audio, and video, which have become essential to tourism activities [6–9]. Meanwhile, artificial intelligence (AI) is creating new possibilities for maintaining lower costs and improving the operational efficiency of interdisciplinary application systems [10]. Recent studies have used AI to automatically recognize tourist UGC image data or text data, thereby effectively reducing the research costs of tourist destination perceptual recognition [11–13]. However, these studies still had several drawbacks despite the progress made. Some studies considered only a single form of data source, failing to combine UGC images, text, and other types of data for analysis, which does not completely consider the integrity of information, resulting in the loss of valuable information [14]. Additionally, studies on the destination perception of tourists mainly focused on one or two of the three dimensions of content perception, sentiment perception, and the perception of spatial and temporal characteristics, failing to combine more dimensions of perception [15–17]. Thus, the completeness of the perceptions is lacking. The perception of different dimensions can represent the destination image and tourist emotion from various aspects, which is beneficial for excavating related tourism elements more profoundly and comprehensively. Additionally, the recognition methods employed in similar research are hindered by their inadequate level of accuracy.

This study proposes an efficient strategy to achieve precise perceptual recognition of tourist destinations while ensuring the integrity of UGC data and the completeness of perception dimensions. This strategy is required to obtain UGC data from online social media platforms and encapsulate the information, such as photos, texts, and geographical coordinates, to form a multi-attribute UGC dataset. Then, we design the improved Inception V3 deep learning model, which utilized the asymmetric convolution and residual functions to replace the original Inception V3 model’s part structure to recognize the UGC dataset’s content perception. Moreover, we integrate the multi-head attention mechanism into the bidirectional long short-term memory (BiLSTM) network and use it to recognize the sentiment perception of the dataset. Statistical processing and geographic information systems (GIS) are used to identify the spatial and temporal characteristics of the dataset. Subsequently, we visualize and analyze the basic tourist feature information from various types of perceptual recognition aforementioned by using a progressive dimension combination method. This method includes one-dimensional, two-dimensional, and three-dimensional perceptual recognition, ranging from independent to cooperative analysis. The recognition results can be used as a valuable reference for destination management decision- making and tourist recommendations.

The article "Multi-dimensional perceptual recognition of tourist destination using deep learning model and geographic information system" was published in 2025. Journal: PLoS One.

The rest of the manuscript is structured as follows:

The Related work section focuses on tourist destination perceptual recognition based on UGC data and introduces deep learning and GIS to tourism research. The Methodology section provides a detailed description of the strategy used. The Experimental results section presents the dataset and recognition results. The Discussion section discusses the significance of the recognition results, the study’s contribution to tourism research, the limitations, and the proposed directions for future studies. Finally, the conclusion is presented in the Conclusions section.

## Related work

### Perceptual recognition of tourist destinations based on UGC data

Exploring tourist destination perception is an important way to represent a destination’s image, explore the destination’s personality, and understand tourist experiences. Afshardoost and Eshaghi [18] conducted a meta-analysis to synthesize the effects of destination images from 87 studies related to destination perception. Polas et al. [19] explored the relationship between destination personality and tourist hesitation through tourist destination perception. Although the studies above have provided an accurate recognition of tourist destination perceptions, the data used have limitations, such as small sample sizes and limited question items. Therefore, their results are subjective.

The increasing number of online social media sites provides a good platform for generating UGC data published online, such as text, photos, audio, and video. UGC data, with their characteristics of low cost, easy access, and high credibility, are becoming more influential in the tourism industry than the information provided by questionnaires and destination marketing organizations (DMOs). The application of UGC data in the tourism industry has emerged as a prominent topic in recent years. Guerrero-Rodriguez et al. [20] analyzed online travel reviews (OTRs) to identify the sentiment perception of a Mexican cultural destination. Liu and Guo [21] used textual data from online travel platforms to represent image perceptions of ice and snow tourism destinations in China. In addition to UGC text data, using UGC image data as unstructured data in travel research is increasing [22]. Image data are more intuitive than text data, and their rich, complex, and powerful communication capabilities are rarely controversial in the tourism industry [23]. For example, Wang, Luo and Huang [24] developed an AI framework to recognize online UGC images and promote people’s understanding of tourism images. Li et al. [25] investigated textual and visual content interaction in online text-photo reviews from Las Vegas tourists and explored tourist sentiment perception. Several studies have also introduced UGC data with geographic information in exploring tourist destination perceptual recognition [26, 27]. However, few of these studies have combined UGC images, texts, and other forms of data for analysis, resulting in a lack of integrity in the research information and ignoring some valuable data. This study encapsulates UGC images, texts, geography, and time data and introduces them into the exploration of tourist destination perception as research materials.

The article "Multi-dimensional perceptual recognition of tourist destination using deep learning model and geographic information system" was published in 2025. Journal: PLoS One.

In recent years, previous studies on tourist destination perceptual recognition have mainly focused on one or two of the three dimensions of content perception, sentiment perception, and the perception of spatial and temporal characteristics. The cognitive experience shapes the tourist experience and the emotions elicited while exploring different attractions [28]. The importance of examining the multi-dimensional information in tourists’ expressions is also proved by relevant research [29]. Therefore, it is necessary to analyze the multi-dimensional perceptions of tourist destinations. Cong, Xu and Fang [30] used UGC travel notes to investigate tourists’ perceptions through content and sentiment analyses, exploring the effect of hosting the Winter Olympics on the image of Beijing’s tourist destination. Some studies have also incorporated spatiotemporal dimensions based on content or sentiment perception [16, 27]. However, few studies have combined more than two perceptual dimensions for cooperative analysis, resulting in a lack of completeness in the perceptual dimension. Based on the abovementioned problems, this study introduces the tourist perception of the destination’s content, sentiment, and spatiotemporal. It combines them into two-dimensional or three-dimensional perceptual recognition for cooperative analysis.

The article "Multi-dimensional perceptual recognition of tourist destination using deep learning model and geographic information system" was published in 2025. Journal: PLoS One.

### Application of deep learning in tourism research

The application of deep learning to mining tourism information has been widely studied in tourism research. Liu et al. [31] used deep learning methods for text classification in the tourism and hospitality field, revealing that deep learning methods are suitable for such tasks. Deep learning models have also been applied in many tourism domains. Table 1 presents some representative studies.

**Table 1:** Review of recent studies relevant to deep learning applied in the tourism domains.

Authors	Research Topic	Method
Han et al. [32]	Daily tourist volume forecasting	A BiLSTM with an attention mechanism was proposed to predict the daily number of visitors to tourist attractions.
Xiao et al. [33]	Tourism destination image	The traditional tourism imagery theory and practice with a visual analysis method were combined based on deep learning to build a relatively complete and a practical research framework for studying tourism destination images.
Su and Yin [34]	Tourism marketing performance evaluation	The superior feature learning capabilities of the ResNet deep learning model were employed to improve the accuracy of the assessment of the actual development of the tourism industry.
Kim, Shin and Kim [35]	Unraveling long-stay tourist experiences and satisfaction	The deep learning-based sentiment analysis was conducted on the 10 identified experience dimensions of long-stay tourists.
Bigne et al. [28]	Exploring the consistency between star ratings and sentiments expressed in online tourism reviews	The recurrent neural network and the long short-term memory (LSTM) was combined and applied to natural language processing.

Based on multiple hidden layers, deep learning models have superior feature learning capabilities, capturing the non-linear relationships between variables, which is one of the crucial reasons for their application in the tourism domain. In addition, deep learning based on computer vision (CV) and natural language processing (NLP) enables quick, accurate recognition and analysis of large amounts of image and text data. A convolutional neural network (CNN) is a representative deep learning model of CV technology that comprises input, convolutional, pooling, fully connected, and output layers. It usually adopts a deep structure, which allows the feature learning of the network to the data, such as images, and stacks up continuously. The feature extraction is sufficient. If the proper weight relation among the neurons in each layer is fitted, the recognition accuracy of the network will be improved. In addition, CNN reduces the number of network parameters and computation costs because of the convolutional kernel weight sharing. These advantages have led to the gradual application of CNNs in the visual analysis of tourist images. Huai et al. [36] used CNN and geo-tagged social media photos to assess the landscape preferences of tourists in urban parks. Razali et al. [37] used a combination of CNN and linear discriminant analysis (LDA) approaches to achieve tourism scene recognition. A recurrent neural network (RNN) is one of the most common neural network units in NLP; it adopts a linear sequence structure and is often used to process sequence information, such as text. The limited context sequence information stored in traditional RNN affects the optimization of network backpropagation, and it is easy to produce the problem of gradient disappearance, leading to a low accuracy of information recognition. As a result, more derivatives of RNN are proposed, such as LSTM, which can capture and transmit a wide range of context information and effectively improve the accuracy of text information recognition. Some studies use the LSTM model or its variants to analyze the sentiment of UGC text review data and to represent implicit semantic features, which is helpful in tourism research [38, 39]. Tourism studies using deep learning in CV and NLP technology are also receiving increasing attention. Bi, Han and Yao [40] integrated CNN and LSTM networks to forecast tourism demand. Meng [41] employed a CNN-BiLSTM model to classify textual data in the smart tourism domain. Wen and Xu [42] used a BERT-BiLSTM-CNN-Attention model to explore the image perception of tourist destinations. Based on the above technical characteristics, this study further improves the classical network model to recognize tourist destination perceptions accurately.

The article "Multi-dimensional perceptual recognition of tourist destination using deep learning model and geographic information system" was published in 2025. Journal: PLoS One.

### Application of geographic information system in tourism research

GIS is a critical spatial information system in tourism planning and spatial analysis. GIS integrates spatial and attribute data and provides functions for processing, storing, analyzing, and visualizing spatial information by combining mathematical methods, remote sensing technology, and database technology. Therefore, some methods, such as kernel density analysis, standard deviation ellipse analysis and hot and cold spot analysis, have been used to characterize tourist spatial perception and movement patterns and explore spatial distribution’s influence on tourism. For example, Ma, Hu and Liu [43] used kernel density and cluster analyses in ArcGIS software to characterize the spatial perception of tourists in island-based tourist destinations. Li et al. [44] recognized the time-space compression effect of the high-speed rail of Chinese tourist destinations using GIS. Zhao et al. [45] used the natural breakpoint grading method and the natural discontinuity point classification method of ArcGIS to divide tourism information flow into different levels. This study adopts the relevant analysis tools of ArcGIS and comprehensively reflects the spatial perception features of tourists to visually recognize the UGC geographic perception data.

## Methodology

### Overall architecture

The overall architecture of the strategy is shown in Fig 1. Different types of UGC data are collected from online social media platforms during the data preparation stage. Then, the data preprocessing involves removing null values, modifying error formats, deleting duplicate data, and other procedures, as described by Wu et al. [46]. After downloading the UGC image data through relevant uniform resource locators (URLs), information such as images, texts, times, and geographical coordinates must be grouped, integrated, and stored in the table of the database system. The final dataset, which includes the multi-attribute UGC data, is used as input for perception recognition, ensuring the information’s integrity. In the stage of perception recognition, an improved Inception V3 deep learning model is proposed to recognize content perception from the UGC dataset. Gradient-weighted class activation mapping (Grad-CAM) is used to validate the performance of the content perceptual model. Grad-CAM, a class-specific localization technique, visualizes the contribution distribution of the CNN-based model’s output via the heat map [47]. Compared to other methods, Grad-CAM offers the advantage of not requiring any modifications to the CNN model structure, facilitating easier deployment. Furthermore, a BiLSTM model with a multi-head attention mechanism is proposed to recognize sentiment perception from the UGC dataset. To identify the perception of spatial and temporal characteristics, we employ statistical processing to count tourist monthly visit frequency and ArcGIS software to achieve relevant recognition. In the visualization and analysis phase, basic tourist feature information, which involves multiple tourist perceptions from the recognition results of the UGC dataset, is visualized and analyzed from a single- or multi-dimensional perspective. We used a progressive combination of dimensions for the perception dimension’s completeness and visualized and analyzed multiple perceptions. In particular, one-dimensional, two-dimensional and three-dimensional perceptions are included in the scope of this study’s method. In the final phase, images of relevant tourist destinations, such as cognitive and affective images, can be represented based on the visualization and analysis results. Based on the research results, we can assist destination managers in making development decisions for local tourism and propose recommendations or suggestions to tourists.

The article "Multi-dimensional perceptual recognition of tourist destination using deep learning model and geographic information system" was published in 2025. Journal: PLoS One.

**Fig 1:** The overall architecture of the strategy.

### Content perception recognition using the improved Inception V3 model

CNN is widely used in image processing tasks such as image classification, target detection, and face recognition. It is also suitable for recognizing content perception from the UGC image data. Based on classical CNN architectures, several open-source CNN variants with higher recognition accuracy and improved performance, such as visual geometry group network (VGGNet), Inception, ResNet, and EfficientNet, have been proposed. The development of large language models has also recently promoted NLP and has provided new methods for image processing [48]. Considering the large language model’s high training cost, the content perceptual recognition model in this study is limited to small or medium sizes. We propose an improved Inception V3 model that replaces the core module structure of the Inception V3 network by applying more asymmetric convolutions and introducing the residual function of ResNet, thereby balancing the width and depth of the network. Furthermore, a dropout layer is added between the global average pooling layer and the fully connected layer so that the neural network units are temporarily dropped from the network with a certain probability during each training iteration. Consequently, it reduces the number of model parameters, alleviating the overfitting problem. Based on the dataset’s size, the model’s complexity, and the degree of overfitting in the training process, the dropout rate is set to 0.3. Moreover, the cross-entropy loss function with label smoothing regularization (LSR) is used in the softmax classification layer, and the noise is added to the one-hot encoded label values, thus reducing the weight of the real sample labels in the calculation of the loss function. This scenario ultimately mitigates the overconfidence of the model [49]. The cross-entropy loss function is calculated as follows:

$$Loss=-\sum_{i}y_{i}logp_{i},$$ (1)

where *p*_*i*_ denotes the probability that the current sample belongs to category *i* and *y*_*i*_ denotes the label value of the sample after one-hot encoding. When the predicted label value coincides with the true value, *y*_*i*_ equals 1; otherwise, it equals 0. LSR adds noise to *y*_*i*_ to obtain *y*_*i*_^*’*^, as follows:

$$\left\{ \begin{array}{c} y_{i}^{\prime }=(1-\varepsilon )*y_{i}+\varepsilon u(N),\\ u(N)=\frac{1}{N}, \end{array}\right.$$ (2)

where *ε* denotes a small positive number, defaults to 0.1, and *N* represents the total number of categories. By introducing *y*_*i*_^*’*^ into the original loss function, the cross-entropy loss function using LSR is obtained as follows:

$$Loss\prime =-\sum_{i}y_{i}^{\prime }logp_{i},$$ (3)

$$Loss^{\prime }=-\sum_{i}[\left(1-\varepsilon )*y_{i}+\varepsilon u(N\right)]logp_{i},$$ (4)

$$Loss\prime =\sum_{i}\{\left(1-\varepsilon )[-y_{i}logp_{i}]+\varepsilon [-u(N)logp_{i}\right]\},$$ (5)

$$Loss\prime =(1-\varepsilon )Loss+\varepsilon \sum_{i}-u(N)logp_{i}.$$ (6)

The complete structure of the improved Inception V3 model is illustrated in Fig 2. InceptionA’ and InceptionC’ depicted in Fig 2 represent the improved Inception modules that replace the original InceptionA and InceptionC blocks, respectively. The details of InceptionA’ and InceptionC’ are illustrated in Figs 3 and 4.

The article "Multi-dimensional perceptual recognition of tourist destination using deep learning model and geographic information system" was published in 2025. Journal: PLoS One.

**Fig 2:** Structure of improved Inception V3 complete model.

**Fig 3:** Structure of improved Inception modules: InceptionA’.

**Fig 4:** Structure of improved Inception modules: InceptionC’.

Fig 3 shows a modification of the InceptionA block module in the Inception V3 model. We replaced the two 3 × 3 convolution layers in the first channel of the original module with two sets of 1 × 3 and 3 × 1 asymmetric convolutions. Concurrently, a residual function was introduced into the asymmetric convolution layer. A skip connection was employed between the two layers to mitigate the vanishing gradient issue arising from the increased depth of the network. This modification also led to a reduction in model parameters. The 3 × 3 convolution layer in the second channel of the original module was replaced with two sets of juxtaposed 1 × 3 and 3 × 1 asymmetric convolution branching channels. The outputs of the branching channels were subsequently feature fused, so obtaining the image information could be more effective by fusing the features extracted from the branch channels. The third and fourth channels agree with the original module. Fig 4 depicts a modification of the InceptionC block module in the Inception V3 model by adding ResNet functions to two sets of 1 × 7 and 7 × 1 asymmetric convolution layers in the first channel of the original module, enabling a skip connection between every two layers, which is also used to alleviate the vanishing gradient issue. The other channels agree with the original module.

The ability of the CNN model should be considered, and the proper training data should be used to improve the accuracy of network recognition. Places365 is an important open-source dataset for scene recognition tasks, containing 1.8 million labeled images from 365 scene classifications that cover most of the real world. Many tourism studies use Places365 to extract the constructed visual symbols of the perceptual imagery of tourist destinations [33]. Based on the characteristics of Places365, such as its large data volume and relevance to tourism, Places365 is selected as the training dataset for the content perceptual recognition model. 365 scene classifications have high scene redundancy for travel tasks, so choosing the most appropriate scenario category from them is necessary. Zhou, Li and Yao [50] discussed that the cognitive image of a destination includes culture, natural landscape, infrastructure, economic environment, natural environment, diet, entertainment, accommodation, social environment, and history. Zhang, Chen and Li [51] classified 12 types of visual content in tourists’ photos. According to the aforementioned studies, the results of content perceptual recognition in our research can be divided into four categories: natural landscape, historical sites, modern urban construction, and civic life. Therefore, 40 scenarios were selected from Places365, each with 5000 training images and 100 validation images, and a total of 204,000 images were used as the final training dataset. The details of categories can be found in Table 2. The representative Places365 images of the 40 scenarios are illustrated in Fig 5.

The article "Multi-dimensional perceptual recognition of tourist destination using deep learning model and geographic information system" was published in 2025. Journal: PLoS One.

**Fig 5:** Representative Places365 images of the 40 scenarios.

**Table 2:** Categories of training dataset for the content perceptual recognition model.

Category	Scenario
Natural landscape	Mountain, valley, canyon, field wild, botanical garden, butte, badlands, river, sky
Historical sites	Temple, pagoda, grotto, museum, ruin, historic site chamber, historic excavation, palace, catacomb, throne room
Modern urban construction	Downtown, transportation facilities, apartment building, aqueduct, factory, plaza, bridge, boardwalk, building facade, construction site
Civic life	Street, crosswalk, bazaar, alley, dining hall, delicatessen, market, banquet, bakery, art gallery, amusement park

To verify the performance of the improved Inception V3 model proposed in this study for content perception recognition, we compared the optimized Top5 recognition accuracies of ResNet34, Inception V3, Resnext50, EfficientNet V2, and the improved Inception V3 models after iterative training using the same Places365 dataset. Top5 accuracy is a metric introduced in the ImageNet competition. In image classification, many objects or scene topics may exist in the image due to the image sources’ uncontrollable photography conditions. If the algorithm predicts an object or scenario that occurs but is not tagged by the training data, the prediction should be considered correct. Therefore, the algorithm should predict the first 5 highest probability results, one of which has been the trained data marked as correct. The image data of the UGC dataset used in this study fit the above situation, so the Top5 accuracy is used to measure the recognition ability of the CNN models. After 100 training episodes, the optimized Top5 accuracies of ResNet34, Inception V3, Resnext50, EfficientNet V2, and the improved Inception V3 model were 88.55%, 95.2%, 90.93%, 88.65%, and 97.8%, respectively. Notably, the improved Inception V3 model exhibited a greater accuracy in this context.

The article "Multi-dimensional perceptual recognition of tourist destination using deep learning model and geographic information system" was published in 2025. Journal: PLoS One.

Based on the above training data and model selection, the process of content perception recognition is as follows:

1. We download the Places365 dataset, and select 40 relevant scenarios, each containing 5,000 labeled training images and 100 labeled verification images.
2. We use the Python PyTorch framework to build an improved Inception V3 network model.
3. Then, we resize the images from the dataset obtained in Step 1 to 299 × 299 × 3 and pass them into the network model for training. After 100 iterations, the content perceptual recognition model is obtained.
4. We apply the content perceptual recognition model from Step 3 to identify and classify the image content in the UGC dataset and obtain the Top5 probability outputs for each image.
5. We use Grad-CAM to visualize and interpret the output of each image.

Grad-CAM uses the gradient of the CNN backpropagation to calculate the weight of the network’s feature layer channel and determine the channel’s importance. Next, a weighted sum of the weights is calculated, and the activation is processed [52]. Finally, important regions are characterized using a heatmap to explain the recognition results. The Grad-CAM core formula is as follows:

$$L_{Grad-CAM}^{c}=RELU(\sum_{k}\alpha_{k}^{c}A^{k}),$$ (7)

where *A*^*k*^ denotes the data for the kth channel in the feature layer, *c* represents the classification category, *α*_*k*_^*c*^ indicates the weight of *A*^*k*^ and *RELU* denotes the activation function.

### Sentiment perception recognition using BiLSTM with a multi-head attention mechanism

NLP is important for achieving speech recognition and text emotion classification tasks. The UGC dataset contains extensive text information, making employing NLP techniques for sentiment perception recognition highly appropriate. In the ecology of NLP, LSTM is an extension of RNN, and it adopts the mechanisms of memory unit, input gate, output gate, and forgetting gate, effectively mitigating the issue of learning long-term dependencies when processing sequence data using an RNN. BiLSTM is a further extension of LSTM that results from a combination of forward and backward LSTMs. BiLSTM is more efficient than RNN and LSTM in capturing bidirectional long-term semantic-dependent information. In addition, the emergence of the attention mechanism strengthens data processing to obtain the attention of different weights. Then, the critical information in the processing object is strengthened, whereas the irrelevant detail information is suppressed. In recent years, a network model combined with the attention mechanism has achieved good performance in NLP [53, 54]. Additionally, the direct use of pre-trained models related to attention mechanisms, such as OpenAI generative pre-trained transformer (GTP) and bidirectional encoder representation from transformers (BERT), for text sentiment analysis is currently an important research method. Still, these models have complex structures and numerous parameters requiring large-scale computing power support. Consequently, we propose a BiLSTM model using the multi-head attention mechanism for recognizing sentiment perception from the UGC dataset, which fully considers the semantic and syntactic connections between sentences and words while controlling the cost of the model and capturing the internal structure of sentences, thereby improving the emotional classification of text. The complete structure of the sentiment perceptual recognition model is illustrated in Fig 6. Based on the dataset’s size, the model’s complexity, and the degree of overfitting in the training process, the dropout rate is set to 0.2.

The article "Multi-dimensional perceptual recognition of tourist destination using deep learning model and geographic information system" was published in 2025. Journal: PLoS One.

**Fig 6:** Structure of the sentiment perceptual recognition model.

The attention mechanism is the multi-head attention mechanism in the transformer model, using a multi-branch self-attention module for parallel computing and integration. In each self-attention module, the query vector Q, key vector K, and value vector V are used to obtain self-attention results. Given the same set of queries, keys, and values, the multi-branch self-attention module provides multiple subspaces, and the model can learn various behaviors based on the same attention mechanism. The different behaviors are then combined as knowledge to extend the model’s ability to focus on different locations. The structure of the multi-head attention mechanism is shown in Fig 7. The *d*^*k*^ in the figure represents the inherent dimension of the self-attention module.

**Fig 7:** Structure of multi-head attention.

After considering the characteristics of web comments in the UGC dataset, the study selected data from Twitter text comments with positive, neutral and negative emotional polarities as the model training and validation data. The performance of the traditional BiLSTM model, the BiLSTM model with a self-attention mechanism, and the BiLSTM model with a multi-head attention mechanism were tested in the same experimental environment based on the above training data. After 100 training episodes, the optimal recognition accuracies of the models were 93.96%, 95.11%, and 98.3%, respectively. The image titles and label text information in the dataset were combined to simplify the recognition process. The process of sentiment perception recognition is as follows:

1. We download data of Twitter text comments with positive, neutral, and negative emotional polarities, each of which is tagged with an emotional polarity. After preprocessing the data, the training and validation datasets are divided in a ratio of 0.85:0.15.
2. We use the Python PyTorch framework to build the aforementioned sentiment perceptual recognition model.
3. The dataset in Step 1 is placed into the model for training, and the trained sentiment perceptual recognition model is obtained after 100 iterations.
4. The model from Step 3 is applied to identify and classify the affective tendencies of the UGC dataset.

### Details of the perceptual recognition of spatial and temporal characteristics

The time information of the UGC dataset may be sparse yearly. Therefore, we employed statistical processing to count the frequency of tourists’ monthly visits and to reflect the temporal recognition results.

The geographic coordinates of the UGC dataset are used to determine the spatial perception of the destination. With the assistance of ArcGIS software, coordinate points can be drawn in map areas for researchers to observe and used in complex spatial analysis using correlation analysis tools, such as kernel density analysis tools. Kernel density analysis is an algorithm used to calculate the spatial distribution of point data and can effectively evaluate the spatial density of point data [55]. The formula is as follows:

$$f(x;\;h)=\frac{1}{nh}\sum_{i=1}^{n}K(\frac{x-X_{i}}{h}),$$ (8)

where *K* denotes the kernel function; *x* signifies the location of the important scenic spots in the destination; *h* denotes the search radius, *X*_*i*_ indicates the spatial location of the sample points in the region formed by the center of *x*, and *n* denotes the total number of sample points. This study uses kernel density analysis tool ArcGIS to recognize the spatial clustering of tourists in the destination.

The article "Multi-dimensional perceptual recognition of tourist destination using deep learning model and geographic information system" was published in 2025. Journal: PLoS One.

### Progressive dimension combination method

A progressive dimension combination method of perceptions is adopted to ensure the completeness of perception dimensions. One-dimensional perception can reflect the basic features of a tourist destination, while two-dimensional perception and three-dimensional perception are used to visualize and analyze the intersection of multiple dimensions. For instance, the sentiment type of the UGC dataset’s content, the spatiotemporal distribution of the UGC dataset’s content, and the spatiotemporal distribution of the UGC dataset’s sentiment should be cross-analyzed to reveal the related tourism elements more comprehensively.

## Experimental results

### Dataset

To examine the performance of the above strategy, we use the UGC data obtained from the Flickr application programming interface (API) to conduct multi-dimensional recognition of the corresponding tourist destinations. Our study area is located in Datong, Shanxi Province, China. Datong is a famous historical and cultural city, with a history spanning over 2,300 years. In particular, many historical sites exist, such as Yungang Grottoes, Xuankong Temple, and the Nine-Dragon Wall. The natural landscape of Datong is rich, such as Heng Mountain, Sanggan River, and soil forest. The abundance of tourism resources makes Datong a suitable case study for tourist destination research.

The data were obtained using the "Flickr.photos.search" method by conducting a fuzzy search with the keywords "Shanxi Datong". Different types of result data were then integrated using photo ID information. The data-cleaning process includes several steps. First, duplicates were identified based on the photo ID, and related data were removed using the "drop_duplicates" method from the "pandas" Python library. Second, data outside the geographic ranges of "39° 54′ –40° 44′ N and 112° 06′ – 114° 33′ E" were discarded. Finally, the data were sorted in chronological order. After data cleaning, we downloaded the photos through the corresponding URLs. We stored the processed UGC photos, along with their associated text, geographic coordinates, time, and other information, in a MySQL database table. The final dataset contains 4,224 records, ranging from 2004 to 2021, with each record including photo ID, photo content, photo title, photo tag, latitude, longitude, and time. Table 3 shows an example of Flickr UGC data from Datong.

**Table 3:** Example of Shanxi Datong UGC data obtained from Flickr.

Photo ID	Photo’s url	Photo’s title	Photo’s tag	Long. and lat.	Take date
50385096657	https://live.staticflickr.com/65535/50385096657_11c9d2cb2e_c.jpg	Datong’s new "old" town centre	Datong shanxi china center centre historical temple pedestrian night iphone dark lights lit	(113.2938, 40.0901)	2020/9/19
46237093581	https://live.staticflickr.com/4899/46237093581_b62476c3b8_c.jpg	Full of people	Asia china shanxi xuankong temple hanging monastery buddhistart landscape dana iwachow daragoman silk road trip 2018	(113.7084, 39.6595)	2018/12/9
28721464895	https://live.staticflickr.com/8724/28721464895_4742b50a69_c.jpg	A smokestack, telling the story of the times, Datong. Gradually closed down a few small coal plants after 20 years	The People’s Republic of China prc China asien asia zhōngguó 2016 chine datong datong shanxi jin shanxi cn china	(113.1675, 40.0344)	2016/8/2
		I don’t know if it will go down like Ruifang, but I’m glad I can see it when it’s busy and grand			

The article "Multi-dimensional perceptual recognition of tourist destination using deep learning model and geographic information system" was published in 2025. Journal: PLoS One.

### Results of one-dimensional perception recognition

We used the recognition models mentioned in the Methodology section to obtain the basic tourist feature information of the dataset. We independently analyzed the one-dimensional recognition of content perception, sentiment perception, and the perception of spatial and temporal characteristics.

Fig 8 shows the results of the content perception recognition. The identified data is the product of the total number of photos and 5 because the Top5 accuracy was used to capture the Top5 most probable recognition results for each photo. Then, the data of various content classifications were displayed in proportions.

**Fig 8:** Results of content perception recognition. A: Group of natural landscapes. B: Group of historical sites. C: Group of model urban construction. D: Group of civic life. E: Overall distribution.

As depicted in Fig 8A, many photos are related to canyons, mountains, valleys, and buttes, which account for 60.74% of the total number of natural landscape photos. This reflects the dominance of the mountain landscape in Datong’s natural landscape. Fig 8B illustrates the recognition of historical sites, mainly focusing on historical site chambers, temples, and catacombs, constituting 15.07%, 14.29%, and 12.39%, respectively. Fig 8C shows the distribution of tourist recognition for modern urban construction. Building facade represents 21.37% of the modern urban construction data, followed by construction sites (16.39%), plazas (11.96%), and bridges (11.90%). As shown in Fig 8D, amusement park comprises the highest proportion (21.49%) of civic life, whereas the percentage of food culture, which local people advocate, is relatively small, with 20.45% of all items in this group. The overall recognition proportion of content perception is illustrated in Fig 8E. The percentage of photos related to historical sites is the highest, at 44.02% of the total, demonstrating that the historical and cultural landscape of Datong is the main tourist attraction. Modern urban construction accounts for 24.55% of the total, followed by natural landscapes that account for 17.67%. However, photos related to civic life are the least, accounting for only 13.75%. Therefore, regarding entertainment, food, and folk culture, the tourist perception of Datong’s offerings seems lacking, indicating a potential oversight in promoting these key tourism elements.

The article "Multi-dimensional perceptual recognition of tourist destination using deep learning model and geographic information system" was published in 2025. Journal: PLoS One.

Fig 9 shows the Top5 classification results of some Places365 verification photos and the visual interpretation of the Top1 results using our code of Grad-CAM technology. As observed from the figure, the Top5 classification results of the first photo are natural landscapes. The area marked by the Grad-CAM thermal map reflects the sky as the main identifying element in the photo. Based on the recognition model of content perception, the second photo’s Top5 probability recognition categories are pagoda, temple, palace, building facade, and apartment building. The Top5 classification of the third photo belongs to the category of modern urban construction, and the Grad-CAM thermal map shows that the building facade is the primary object identified. The classification results of the last photo are related to the lives of the citizens and focus on the food culture, which agrees with the content of the photo. Fig 9 also illustrates the high accuracy and good interpretability of the recognition model of content perception and the Grad-CAM visualization technique.

**Fig 9:** Top5 classification results of Places365 verification photos and Grad-CAM visualization of the Top1 results.

The UGC textual data of the dataset are classified into positive, neutral, and negative emotional tendencies using the recognition model of sentiment perception. The amount of data with neutral sentiments is 1,827, followed by positive and negative sentiments, which are 1560 and 837, respectively. Based on further artificial examinations, UGC textual data classified as positive emotional tendencies usually contain words such as "Love" and "Beautiful." The data classified as neutral emotional tendencies do not have apparent positive or negative emotional words. The data classified as negative emotional tendencies contain "Hate" and "Cold." The results obtained from the recognition model of sentiment perception demonstrate that the perception of tourist sentiment in Datong is mainly neutral. Moreover, positive sentiment occupies a high proportion, and the quantity is close to neutral sentiment. Although the negative sentiment is the lowest number, its corresponding number exceeds half that of the positive sentiment data. Some representative words for each emotional tendency are illustrated in Table 4.

The article "Multi-dimensional perceptual recognition of tourist destination using deep learning model and geographic information system" was published in 2025. Journal: PLoS One.

**Table 4:** Representative words of emotional tendencies.

Emotional Tendency	Representative Words
Positive	Love, beautiful, magnificent, good, nice, lovely, delicious, happy
Neutral	Strange, formal, new, normal, obvious
Negative	Hate, cold, full of people, lonely, sad

Based on the time information of the UGC data, we obtain the frequency change curve of the dataset, as depicted monthly in Fig 10. The figure shows that the data volume fluctuates significantly with the monthly change, demonstrating the seasonal shift in tourist time perception in Datong. Notably, the UGC data volume reached its lowest in January, with only 17 records. From February to May, the increase in data volume is particularly noticeable, revealing a strong correlation between time perception and warmer weather. The data decrease rapidly in June, suggesting the possible influence of the lower number of statutory holidays that month. From July to September, the volume of UGC data increases significantly, with 656, 731, and 715, respectively. Subsequently, it decreases in October, from 715 to 374. Then, the data volume increases slightly in November and decreases to 150 in December. Overall, tourists perceived the most information in the summer and the least in the winter.

**Fig 10:** Changing the process of temporal perception.

To identify the spatial perceptions of the experimental datasets, such as spatial distribution and spatial kernel density, we utilized the ArcGIS software tool to analyze the spatial characteristics of the data. The output pixel size of kernel density analysis is set to 0.001; the gradient class number is 30, and the method of data resampling type is "Cubic." As depicted in Fig 11, the kernel density mapping results reveal that tourists are primarily concentrated in three areas, represented by three red circular patterns. From left to right in Fig 11, the three red circular patterns represent three tourist attractions: Yungang Grottoes, Datong Ancient City, and Heng Mountain. Among them, Datong Ancient City is the most densely visited area. This is because of its rich historical sites, including Huayan Monastery, Fahua Temple, and Prince Dai Residence. Yungang Grottoes is second only to Datong Ancient City in terms of the degree of spatial perception clustering among tourists. Yungang Grottoes, a world heritage site and one of the 5A tourist attractions of China, always attracts numerous tourists. 5A tourist attractions in China often have national or world-class natural and cultural heritage, representing the highest level of Chinese tourist attractions. 4A tourist attractions in China also have rich tourism resources, but they may lack the national or world-class exclusivity of 5A sites. Based on the kernel density mapping results, Heng Mountain is ranked third. The mountain is a renowned 4A tourist attraction in China, with its fame dating back to ancient times.

The article "Multi-dimensional perceptual recognition of tourist destination using deep learning model and geographic information system" was published in 2025. Journal: PLoS One.

**Fig 11:** Spatial perception of Datong. Reprinted from Big Data Institute of Shanxi Datong University under a CC BY license, with permission from Big Data Institute of Shanxi Datong University, original copyright 2024.

### Results of two-dimensional perception recognition

The combination of multi-dimensional perception recognition analysis can be a fine-grained representation of the tourism destination situation. As a result, we combine the two types of perceptual dimension recognition data to show the synergistic effects among the dimensions. The combination of content perception and sentiment perception was used as an example.

Table 5 illustrates the sentiment distribution for each type of content perception data, and the content perception data are classified based on the Top5 accuracy, so the total number of data points in the table is 21,120. Through observation and analysis of the emotional tendencies corresponding to the four types of content perception, it was found that the ratio of positive and neutral samples (positive and neutral emotional tendencies) to negative samples (negative emotions) is the largest at 6.11 in historical sites. Fig 8E shows that historical sites account for the highest proportion (44.02%) of overall content perception. Therefore, it is possible that when attention to tourist sites is high, the corresponding tourist emotional tendency is more likely to be positive. Additionally, the ratios for natural landscapes, modern urban construction, and civic life are 3.02, 2.81, and 3.95, respectively. Given the low proportion of these types of content perceptions within the overall content perception distribution, it is difficult to establish a clear relationship between the degree of attention to the content and tourist emotional tendencies. The detailed data volume of emotional tendencies based on 40 scenarios can also be found in Table 5. There are far more positive emotions than negative emotions in all scenarios of historical sites. The positive and negative emotions in most civic life scenarios are close to each other, showing how polarized the comments are. Additionally, we can find some scenarios of natural landscape, such as butte and badlands, and model urban construction, like factory and boardwalk, with more negative emotional tendencies than positive emotional tendencies.

The article "Multi-dimensional perceptual recognition of tourist destination using deep learning model and geographic information system" was published in 2025. Journal: PLoS One.

**Table 5:** Volume of content perception corresponding to emotional tendencies.

Classification of content perception	Positive	Neutral	Negative
Natural landscape	1,293	1,515	930
Mountain	258	362	89
Valley	113	208	97
Canyon	284	315	165
Field wild	66	82	53
Botanical garden	92	73	80
Butte	103	164	112
Badlands	63	91	164
River	144	167	122
Sky	170	53	48
Historical sites	3,823	4,163	1,307
Temple	416	725	187
Pagoda	276	327	167
Grotto	125	414	94
Museum	264	326	118
Ruin	388	428	163
Historic site chamber	625	617	158
Historic excavation	147	523	100
Palace	433	393	133
Catacomb	763	286	104
Throne room	213	124	83
Model urban construction	1,873	1,959	1,364
Downtown	112	114	75
Transportation facilities	103	69	55
Apartment building	186	197	124
Aqueduct	108	183	74
Factory	81	83	83
Plaza	198	254	169
Bridge	272	241	105
Board walk	73	112	160
Building facade	354	433	323
Construction site	386	273	193
Civic life	811	1,498	584
Street	82	131	73
Crosswalk	75	103	53
Bazzar	84	61	58
Alley	68	218	66
Dining hall	17	23	9
Delicatessen	80	71	74
Market	81	108	47
Banquet	9	11	5
Bakery	107	126	60
Art gallery	121	184	66
Amusement park	87	462	73

### Results of three-dimensional perception recognition

We combine three perception dimensions to make the visualization display of recognition and make the representation of the perception result more cooperative. This study cross-analyzes the spatiotemporal distribution of content perception and sentiment perception.

The content perception recognition data are divided by quarters, and the spatial visualization of the data is achieved by combining the geographic information (Figs 12–15). As illustrated in Figs 12–15, the circular pattern represents the perception data of natural landscapes, the rectangle pattern represents the data of historical sites. The triangular pattern represents the data of modern urban construction, and the diamond pattern represents the data of civic life. Fig 12 shows the spatial distribution of content perception recognition data for the first quarter (January–March), with the lowest data volume for the four quarters. The data distribution is mainly concentrated in Yungang Grottoes, Datong Ancient City, and Heng Mountain. Data for other areas are particularly scarce. In these three tourist attractions, the spatial superposition of different types of content perception data reflects the diversity of the tourist content perceptions of the core scenic spots. Fig 13 illustrates the spatial distribution of the data for the second quarter (April–June). The three core tourist attractions’ impact areas are spread during the second quarter. In addition, in the central part of Datong, data collection areas are dominated by natural landscapes, historical sites, and modern urban construction. This reveals that the number and area of regions where tourists have a high content perception level increases with the geographical space’s warming climate. Moreover, because of the larger volume of data in the third quarter (July–September), there are more areas of content perception. As depicted in Fig 14, the area of influence and interest of the core scenic areas has expanded further. Owing to the adjacency of the Yungang Grottoes and Datong Ancient City, the area between these two scenic spots is connected by content perception data, forming a larger data aggregation area. Additionally, the northern area of Datong Ancient City appears to be connected to the zonal content perception data aggregation area of Inner Mongolia, indirectly indicating that cross-provincial tourism concerns influence each other. In the fourth quarter (October–December), content perception attention decreases significantly, with a significant reduction in data aggregation areas, as shown in Fig 15. Overall, many types of data are in the spatial overlay of content perception data, and a single type of content perception data rarely forms an aggregation in the space. This is more evident within the geographical scope of the core scenic spots. There is a high probability that regions between the core scenic spots are influenced by the scenic spots to form content perception data aggregations, which may be linked to the core scenic spots in the peak season.

The article "Multi-dimensional perceptual recognition of tourist destination using deep learning model and geographic information system" was published in 2025. Journal: PLoS One.

**Fig 12:** Spatiotemporal distribution of content perception (January to March). Reprinted from Big Data Institute of Shanxi Datong University under a CC BY license, with permission from Big Data Institute of Shanxi Datong University, original copyright 2024.

**Fig 13:** Spatiotemporal distribution of content perception (April to June). Reprinted from Big Data Institute of Shanxi Datong University under a CC BY license, with permission from Big Data Institute of Shanxi Datong University, original copyright 2024.

**Fig 14:** Spatiotemporal distribution of content perception (July to September). Reprinted from Big Data Institute of Shanxi Datong University under a CC BY license, with permission from Big Data Institute of Shanxi Datong University, original copyright 2024.

**Fig 15:** Spatiotemporal distribution of content perception (October to December). Reprinted from Big Data Institute of Shanxi Datong University under a CC BY license, with permission from Big Data Institute of Shanxi Datong University, original copyright 2024.

Figs 16–19 illustrate the spatial visualization of the three types of sentiment perception data in various quarters. As depicted in Figs 16–19, the circular pattern represents the perception data of positive emotional disposition; the rectangle pattern represents the data of neutral emotional disposition, and the triangular pattern represents the data of negative emotional disposition. As shown in Fig 16, different types of emotional polarities may exist in the same geographical location, demonstrating that tourist sentiment perception has obvious individual characteristics. In addition, the three core scenic spots in Datong in the first quarter have mainly positive and neutral emotions, and the distribution of negative emotions is relatively independent and scattered around the core scenic spots. As illustrated in Fig 17, numerous neutral and negative emotional areas account for a large proportion of non-core scenic spots, indicating that the development of scenic spots is unbalanced, and the user experience of non-core scenic spots quite differs from that of core scenic spots. Although the sentiment perception of visitors increases in the second quarter, there is a corresponding increase in negative emotions. The warm season increases visitors’ attention, but the positive effect on the experience is unobvious. As illustrated in Fig 18, the proportion of negative emotions in non-core scenic spots is further expanded, especially in central and eastern Datong, where negative emotions exceed positive emotions, highlighting scenic areas related to poor user experience and other issues. As depicted in Fig 19, neutral emotion is dominant and negative emotion is stable in the fixed region. Comprehensive analysis demonstrates that in Datong, seasonal climate change affects tourist-perceived attention. Still, the effect on emotional polarity is unobvious, and the emotional polarity of scenic spots is relatively stable.

The article "Multi-dimensional perceptual recognition of tourist destination using deep learning model and geographic information system" was published in 2025. Journal: PLoS One.

**Fig 16:** Spatiotemporal distribution of sentiment perception (January to March). Reprinted from Big Data Institute of Shanxi Datong University under a CC BY license, with permission from Big Data Institute of Shanxi Datong University, original copyright 2024.

**Fig 17:** Spatiotemporal distribution of sentiment perception (April to June). Reprinted from Big Data Institute of Shanxi Datong University under a CC BY license, with permission from Big Data Institute of Shanxi Datong University, original copyright 2024.

**Fig 18:** Spatiotemporal distribution of sentiment perception (July to September). Reprinted from Big Data Institute of Shanxi Datong University under a CC BY license, with permission from Big Data Institute of Shanxi Datong University, original copyright 2024.

**Fig 19:** Spatiotemporal distribution of sentiment perception (October to December). Reprinted from Big Data Institute of Shanxi Datong University under a CC BY license, with permission from Big Data Institute of Shanxi Datong University, original copyright 2024.

### Comparison results of model accuracy

To verify the accuracy of the content perceptual recognition model in a specific application scenario, we conducted an accuracy comparison experiment of content perception among the various models. We used the method of artificial judgment of the Top1 and Top5 categories to label 4,224 tourist UGC images in the Datong dataset, We considered this model artificial judgment result as the basis for comparison. Then, the UGC images were recognized using the model proposed in this study, and the ResNet34, Inception V3, Resnext50, and EfficientNet V2 models. If the Top1 category predicted from the recognized image was the same as the artificial judgment Top1 category, the Top1 recognition result was considered accurate. If any of the Top5 categories predicted from the recognized image overlapped with the artificial judgment Top5 categories, the Top5 recognition result was considered accurate. The recognition accuracy results are shown in Table 6, revealing that our model has the highest accuracy in the Top1 and Top5 categories at 0.8078 and 0.9839, respectively.

**Table 6:** The Top1 and Top5 accuracy of content perception recognition using various models.

Models	Resnet34	Inception V3	Resnext50	EfficientNet V2	Improved Inception V3
Metric					
Top1 accuracy	0.6792	0.7924	0.7907	0.7069	**0.8078**
Top5 accuracy	0.8648	0.9448	0.9384	0.9181	**0.9839**

To verify the accuracy of the sentiment perceptual recognition model in a specific application scenario, we conducted an accuracy comparison experiment of sentiment perception among different models. We used the method of artificial judgment of emotional polarity to label 4,224 tourist UGC texts in the Datong dataset and considered this artificial judgment result as the basis for comparison. Then, the UGC texts were processed using the model proposed in this study, the traditional BiLSTM model, and the BiLSTM with a self-attention mechanism. The prediction was considered accurate if the recognition was consistent with artificial judgment. The comparison results are illustrated in Table 7. Our model showed the highest accuracy (0.9742) among the three models.

**Table 7:** The accuracy of sentiment perception recognition using various models.

Models	BiLSTM	BiLSTM with a self-attention mechanism	BiLSTM with a multi-head attention mechanism
Metric			
Accuracy	0.9112	0.9505	**0.9742**

## Discussion

The perceptual recognition models used in the strategy exhibit an exact identifying ability to characterize the content or sentiment from the UGC dataset. The accuracy of the proposed models is higher than that of the compared models Whether in the training stage of the models or the application of the experimental case. For content perception recognition, the Top5 accuracy of the proposed model was 97.8% in the training stage, and its Top1 and Top5 accuracies were 80.78% and 98.39%, respectively, in the experiment. In contrast, other related studies did not achieve a Top5 accuracy above 97% [11, 23, 26]. For sentiment perception recognition, the accuracy of the model was 98.3% in the training stage and 97.42% in the experiment. The proposed model shows better recognition accuracy than those of other related studies [53, 54]. In addition, the Grad-CAM visualization of content perception and the artificial examination of sentiment perception proved that the recognition models were effective. Furthermore, the strategy mainly provides a model-agnostic framework. The recognition models used in this study can be replaced by other models if there is a need for better alignment with the application scenario.

The article "Multi-dimensional perceptual recognition of tourist destination using deep learning model and geographic information system" was published in 2025. Journal: PLoS One.

Multi-attribute UGC data, including images, texts, time, and geographic information, are adopted as the input for tourist destination recognition, providing an opportunity to use UGC information integratively and collaboratively. Similarly, the rapid development of multi-modal machine learning has proven the importance of taking advantage of the correlations and complementarities between different types of data [56]. With support from online social media platforms, access to data has become easier and the volume of available data has increased. Consequently, using multi-attribute data is no longer a challenge. In our experiment, a sufficient amount of data can be obtained even though the study area, called Datong, is an ordinary city with a ranking of approximately 100 in the Chinese city ranking list.

Compared with previous studies, this study considers the completeness of the perceptual dimensions more fully. The progressive dimension combination method of perceptions, which involves one-dimensional, two-dimensional, and three-dimensional perceptions, is adopted. One-dimensional perception recognition is used to achieve independent analysis and then to characterize the basic features of a tourist destination. Based on the one-dimensional perception recognition results, it is obvious that the historic city features of Datong are the most attractive to tourists and are the main tourist elements of Datong. Although there are local traditional foods, entertainment, and other rich elements of civic life in Datong, tourists take the lowest proportion of relevant photos, and folk customs in visual projection are ignored. From a sentiment perspective, the emotional tendency of tourists toward Datong is mainly positive and neutral, but many tourists still show negative emotions. The time perception of tourists in Datong follows a pattern: the higher the temperature, the greater the frequency of visits. Summer has the most visits, whereas winter has the least. Datong is located in the northern inland region of China, and the summer climate is cool and comfortable, making it suitable for tourism and vacations. Winter is cold and dry, resulting in a corresponding decrease in tourism. Regarding spatial perception, tourists mainly gather in Datong Ancient City, Yungang Grottoes, and Heng Mountain.

The article "Multi-dimensional perceptual recognition of tourist destination using deep learning model and geographic information system" was published in 2025. Journal: PLoS One.

The data distribution in other areas is very sparse, indicating a highly uneven spatial distribution of tourism popularity. Two-dimensional and three-dimensional perception recognitions are utilized to achieve collaborative analysis, thereby elucidating the relationship between different dimensions of perception and unveiling the related tourism elements more deeply and comprehensively. This study explored the sentiment distribution within content perception data and revealed a positive correlation between the perception of tourist content and sentiment towards Datong. When attention to content perception approaches approximately half of the total data volume, a positive correlation is observed between positive emotion and content perception. The spatial and temporal distributions of content perception are also demonstrated. In the case of Datong, numerous types of data are superimposed within the spatial dimension of content perception, a phenomenon that is particularly pronounced in core scenic spots. In contrast, it is difficult for a single category of content perception data to constitute a spatially cohesive region. With the change in time, in the peak season of tourism, the attention of the core scenic area is further expanded, showing the tendency of spreading to the outside of the scenic area in the geographical space, which achieves the convergence of the geographical space of the core scenic area; this conclusion basically agrees with the results of previous studies [57, 58]. Moreover, during the peak season, Datong and its adjacent regions in Inner Mongolia exhibited belt-shaped areas of aggregated content perception data aligning with the pattern of intercity tourism economic ties in the Yellow River basin, as explored by Zhang et al. [59]. The study also analyzed the spatial and temporal distribution of the sentiment perceptions of tourists in Datong and found that different types of emotional polarities existed in the same geographical location. The sentiment perception of tourists exhibits obvious individual characteristics. The emotional polarity of each scenic spot is relatively stable. Positive and neutral emotions are predominant emotions in the core scenic spots, whereas negative emotion is relatively more prevalent in the non-core scenic spots.

The article "Multi-dimensional perceptual recognition of tourist destination using deep learning model and geographic information system" was published in 2025. Journal: PLoS One.

The recognition results can be used to explore images of tourist destinations. The image of a tourist destination is an aggregation of tourist thoughts, emotions, and impressions of the destination. The models mentioned in our strategy can identify visual information from photos and sentiment information from texts. In addition, the spatial and temporal distributions of tourist information can be represented using this strategy. Therefore, the methods presented are suitable for studying tourism destinations. Another important use of the recognition results is to provide a basis for making suggestions to destination managers and tourists. In our experimental case, we provide the following suggestions for destination managers and potential visitors to Datong: (1) Destination managers should intensify their efforts to create awareness about the civic life of the content perception category. For instance, tourism marketing should focus on promoting food products and other content displays to foster the creation of diversified tourism and cultural offerings, such as fast-food knife noodles, paper-cut crafts, and other attractions. Additionally, they should optimize the spatial layout of facilities related to civic life, integrate the spatial structure with the analysis of tourist gaze behavior, and suitably develop unexplored tourist areas. (2) Destination managers should enhance the infrastructures and services of relevant scenic spots, which includes constructing more tourist centers using a humanistic approach, emphasizing the experiential needs of tourists, and developing precision marketing strategies. When designing travel routes, destination managers should consider the varying preferences of tourists and attend to differences in their needs. (3) It is necessary to further develop potential tourism resources in the northern and southern parts of the city, enhance the transportation network within and between scenic spots, and bolster connectivity among them. Additionally, attention should be paid to developing provincial scenic spots alongside new and diversified types of content-rich tourist attractions. (4) It is recommended that potential visitors travel to Datong during the summer to make the most of the season and avoid winter travel. The results can be used as multi-modal basic input data for the tourism recommendation system.

The article "Multi-dimensional perceptual recognition of tourist destination using deep learning model and geographic information system" was published in 2025. Journal: PLoS One.

The main contributions of this study are as follows:

1. We propose a strategy that can achieve precise perceptual recognition of tourist destinations while ensuring the integrity of UGC data and the completeness of perception dimensions. This strategy combines deep learning, tourist perception, spatial geography, and other disciplines to improve the efficiency of data identification and analysis. From the perspective of tourism theory construction, it offers a methodological approach to perception research in tourism destinations and serves as a practical reference for exploring the tourism industry.
2. We introduce an improved Inception V3 model for content perception recognition, employing asymmetric convolution and residual functions to balance the width and depth of the network, alleviating the overfitting problem and achieving a more accurate identification of visual information. Additionally, we integrate the multi-head attention mechanism into the BiLSTM model for sentiment perception, fully considering the semantic and syntactic connections between sentences and words while controlling the cost of the model.

This study has several limitations. First, the strategy does not incorporate the recognition and analysis of UGC video content. This omission neglects the potential insights from mining dynamic visual materials using storylines. Second, recognition tasks currently require the use of multiple models. It would be more efficient if a single model could recognize basic information, such as content and sentiment perception. Third, having a larger data volume for the case study is better, as this can improve the analysis efficiency. Based on the framework of the strategy discussed, future research will consider the encapsulation of UGC video data into the multi-attribute UGC dataset, and researchers will utilize large language model technology to develop a tourism perception recognition model with multi-modal input and output, thereby replacing the current multiple models. In addition, we will apply the recognition results to develop a personalized tourism recommendation system by utilizing them as fundamental data to address issues such as the cold start problem.

## Conclusions

This study proposed an effective strategy for achieving the multi-dimensional perceptual recognition of tourist destinations. The multi-attribute UGC dataset was utilized as the input data, ensuring the integrity of tourist information. A progressive dimension combination method was adopted to ensure the completeness of the perception dimensions. The models exhibit high recognition accuracy. The recognition results can be used to represent the image of the tourist destination and can also provide decision-making assistance for destination managers and potential tourists. This study provides an essential reference for a tourist destination’s methods and research route selection. Its application can be extended to future research on personalized tourism recommendation systems.
